# Deep Transfer Learning for Question Classification Based on Semantic Information Features of Category Labels

**DOI:** 10.1155/2022/7178818

**Published:** 2022-09-30

**Authors:** Lei Su, Wenqian Kang, Liping Wu, Di Jiang

**Affiliations:** School of Information Engineering and Automation, Kunming University of Science and Technology, Kunming 650504, China

## Abstract

Question classification is an important component of the question answering system (QA system), which is designed to restrict the answer types and accurately locate the answers. Therefore, the classification results of the questions affect the quality and performance of the QA system. Most question classification methods in the past have relied on a large amount of manually labeled training data. However, in real situations, especially in new domains, it is very difficult to obtain a large amount of labeled data. Transfer learning is an effective approach to solve the problem with the scarcity of annotated data in new domains. We compare the effects of different deep transfer learning methods on cross-domain question classification. On the basis of the ALBERT fine-tuning model, we extract the category labels of the source domain, the question text, and the predicted category labels of the target domain as input to extract the category labels. Additionally, the semantic information of the category labels is extracted to achieve cross-domain question classification. Furthermore, WordNet is used to expand the question, which further improves the classification accuracy of the target domain. Experimental results show that the above methods can further improve the classification accuracy in new domains based on deep transfer learning.

## 1. Introduction

Question classification plays a vital role in the quality and performance of the QA system, which can restrict answer types, accurately locate and verify answers, and provide information and conditions for the answer selection strategy. For example, question “what differentiate between force and momentum” is mainly about getting an answer about science, rather than searching for social, economic, educational information. The answer should be consistent with the category of the question, so it is only necessary to focus on the “science” domain in the answer extraction stage. Early question classification uses a rule-based method [1, 2], attempting to match the question with manually defined rules and high labor costs. Sangodiah et al. [3] proposed a novel feature type based on taxonomy with a support vector machine (SVM) to improve the accuracy of question classification for data sets having questions from various fields. Silva et al. [4] combined a rule-based method with a machine learning-based method.

The main problems with traditional classification methods are as follows: the text representation having a high latitude and a high sparseness, weak feature expression ability, requirement of manual feature engineering, and high cost. Deep learning automatically obtains features by using CNN [5, 6], RNN [7, 8], LSTM [9, 10], and other network structures, subtracts complicated artificial feature engineering, and realizes an end-to-end solution. However, due to the strong dependence of deep learning on manually labeled data, it brings problems, such as insufficient training data and a weak interpretability of the model. Moreover, when deep learning models are used during NLP tasks, they are all based on the fact that the training data and the test data have a common feature space and the same data distribution and cannot meet the question classification in different domains. Therefore, the question classification model is constructed by the existing related source domains to extract relevant shared knowledge, and it is applied in the new domain to reduce the dependence on artificially labeled data when constructing the question classification model in the new domain. Li et al. [11] proposed a novel approach named topic correlation analysis (TCA), which extracts both the shared and the domain-specific latent features to facilitate effective knowledge transfer.

Transfer learning is an effective solution for a scarcity of labeled data, which entails transferring the related tasks and knowledge of other scenes that have been mastered to new scenes to adapt to new tasks and learn new knowledge. In recent years, transfer learning has achieved substantial growth in QA systems, such as question classification, semantic analysis, and question-answer matching. In the question classification scenario, we only consider domain adaptation [12] with different domains, but it is still the same task. Transferred component analysis (TCA) [13] attempts to map the data of the source domain and the target domain in reproducing kernel Hilbert space (RKHS) [14]. Then, maximum mean discrepancy (MMD) is used to minimize the distance between the two domains with an average accuracy in the text classification experiment of 0.6865. Joint distribution adaptation (JDA) [15] adapts the marginal distribution and the conditional distribution of the source and target domains at the same time, though the classification effect is better than TCA.

Yosinski et al. [16] studied whether deep neural networks can be transferred. They proposed a method to measure the versatility and specificity of different layers of deep learning networks to determine the degree of which the features of the layer can transfer from one task to another. Howard and Ruder proposed an efficient transfer learning method for any task in NLP, which is the Universal Language Model Fine-Tuning (ULMFIT) [17]. ULMFIT first pretrains the language model (LM) and then fine-tunes the language model and finally the classification task. Although ULMFIT can learn the relationship between contexts, it cannot be parallelized, which makes model training and inference difficult. A transformer [18] models the context by self-attention, increasing the speed of training and inference. Devlin et al. [19] proposed a transformer encoder-based pretrained model, BERT, which directly learns the contextual information of the text. Additionally, it is more efficient and captures longer-distance dependencies than RNN in 11 natural language processing tasks. In 2020, Zhen et al. [20] proposed the ALBERT model to reduce memory consumption and improve training speed.

The above transfer learning method extracts features from the training text, ignoring the semantic information provided by the text label. For example, the source domain question set contains labels such as “sport” and “family,” and these labels themselves carry semantic information [21–23]. Therefore, if we use the semantic information of these labels for training the classifiers, we compare the semantic similarity of the labels and the ask statements, before obtaining an association of the two. Then, when extending the classifier to the target domain where the classes are “culture” and “society,” we can predict the association between the questions and the labels while obtaining the semantic information of the target labels. This improves the accuracy of the classification predictions for new categories in different domains.

Therefore, this study proposes inputting the question text and the prediction category label containing semantic information into ALBERT for fine-tuning and decomposing the classification problems into general bi-classification (true/false) to output true/false prediction results. We refer to this as L-ALBERT-FiT (a question classification method based on deep transfer learning and semantic information features of category labels). Experimental results show that the classification accuracy of L-ALBERT-FiT is improved by approximately 3.73% compared to the BERT fine-tuning model and approximately 5.92% compared to the ALBERT fine-tuning model. Furthermore, we expand the synonyms of the question dataset, increase the feature extraction and further improve the classification accuracy of the question. The accuracy of question classification is very important to the overall performance of the question answering system.

Section 2 introduces the basics required for this study, including deep transfer learning and labeling semantic information.  Section 3 describes the question classification method based on deep transfer learning and semantic information features of category labels.  Section 4 verifies the validity of the proposed model using comparative experiments. Finally, a summary of the full text is presented.

## 2. Related Work

Pan et al. [13] applied TCA to domain adaptation (DA) and implemented cross-domain text classification. TCA uses MMD learning transfer components, making the data distribution similar in different domains in these transfer components according to the distribution measure of RKHS [14]. Subsequently, Long et al. [15] proposed JDA, which gradually improves the accuracy of pseudo-labels by sampling repeated iterations. Howard and Ruder [17] used the language model AWD-LSTM [24] for transfer learning in text classification. ULMFIT considerably outperforms CoVe, oh-LSTM, Virtual, CNN, and DPCNN on six text classification tasks, and the test error rate is the smallest. Akbik et al. proposed Flair [25], a sequence tagging architecture based on neural language modeling, which implemented a series of classic NLP tasks (such as named entity recognition (NER) and partial entities) and set up state-of-the-art technology to score speech (POS tagging). Flair's method of extracting contextual string embedding from character-level language models can be used to build text classifiers.

BERT [19], as a deep transfer model, uses a transformer as the main framework to substitute word2vec for 11 NLP tasks, such as text classification. The two steps of BERT's work are first to initialize the pretrained parameters and then to fine-tune the parameters based on the data from the downstream task. Different downstream tasks have their own fine-tuning models. Chi Sun et al. [26] compared the performance of different fine-tuning methods of BERT on text classification. BERT's pretraining objectives are autoencoding (AE), and in the fine-tuning stage, without the MASK, it causes inconsistent pretraining and fine-tuning data, thus introducing some human error. XLNet [27] uses the AR model to replace the AE model, which solves the negative effects of the MASK. Since the AR model is unidirectional and cannot predict targets based on context relationships, XLNet [27] uses all possible permutations to maximize the expected log likelihood of the factorization order of all possible sequences. For noise reduction and automatic encoding preprocessing, BERT performs better than XLNet. However, BERT ignores the dependence between masked positions and has problems, such as pre-fine-tuning differences, which XLNet can address and overcome the limitations of BERT. In the experiments, it was found that XLNet is more effective when reading comprehension tasks of long texts. BERT tends to expand the model size when processing downstream tasks, and the training time is lengthened due to processor memory limitations. To solve these problems, Lan et al. proposed a technology that reduces memory consumption and improves BERT's training speed-ALBERT [20]. ALBERT uses factorization to reduce the number of parameters of the embedding mapping module and shares the parameters between layers. On the pretraining task, ALBERT strengthens the continuity of the network learning sentences while removing dropout layers. Dropout has a notable effect in preventing overfitting. However, MLM is difficult to overfit. Removing dropout layers can free up much memory occupied by temporary variables, which improves the memory. Overall, ALBERT's contributions include improving parameter efficiency, improving self-supervised learning tasks, increasing the capacity of the model, and increasing the scale of the training data.

Traditional question classification methods ignore the semantic information provided by natural language labels. The class labels carry semantic information itself [21–23]. If we want to extend the classifier to another class with only a few training examples, we can use the semantics provided by the category labels. Puri and Bryan [22] took the natural language describing the classification task as an input and the natural language answer was obtained after the model was trained. Halder et al. [23] proposed a zero-shot learning method, task-aware representation of sentences (TARS). TARS factorizes any classification problem into a general binary classification problem and injects the concept of the task itself into the transformer model to preserve the two abovementioned pieces of information and then improve the classification effect. TARS has a higher classification accuracy rate in the domain of sentiment analysis but a lower classification accuracy rate in question and topic types. Zhang et al. [28] proposed a universal domain adaptation method for fault diagnosis. The proposed method achieves cross-domain fault diagnostics prediction without explicit assumptions made on the target label set.

## 3. Methods

Given the strong generalization and feature extraction capabilities of deep transfer learning, this study proposes a question classification method based on deep transfer learning and semantic information features of category labels, which consists of 3 parts.

### 3.1. Model Transfer

As shown in Figure 1, we first compose all of the labels of the source domain and the target domain into a label dictionary. The source domain question is used to train the model and all of the labels in the label dictionary are generated as one-to-one corresponding input tuples <label, question>, and the tuples are input into the L-ALBERT-FiT model. Second, the model extracts the semantic information of the category label and compares the semantic similarity of the label and the question to obtain the relevance of the two. Then, when this classifier is extended to the target domain for classification, we obtain the target domain label's semantic information under the premise, and the relevance of the question and label can be predicted. Finally, the L-ALBERT-FiT is fine-tuned with a small amount of target domain data and the linear output layer of the ALBERT is replaced with a TRUE/FALSE selection to predict the question classification results. As a result, the scarcity of the annotated questions for new domain categories could be solved.

As shown in Figure 1, L-ALBERT-FiT is trained on the source domain and is fine-tuned in the target domain. We input a few target domain samples into the pretrained model and fine-tune part of the parameters of the model in the process of retraining the model. Finally, the target domain question was inputted to test the transferability of L-ALBERT-FiT.

We generate a label dictionary with the class labels of the source domain and the target domain to provide the label dictionary to L-ALBERT-FiT as an additional input. This means that we add the semantic information of the class label to the question sentence while extracting the features of questions and labels, before discovering the connection between the labels and sentences. For example, as shown in Figure 2, the label dictionary generated by the source and the target domain contains the labels “sports”, “relationships”, “computer”, and “finance”, and we enter the question “who is the best football player in Europe to date?” into the model. Then, the input data includes the questions and possible labels, while the tuples are entered as follows: <“sports”, “who is the best football player in Europe to date”> <“relationships”, “who is the best football player in Europe to date”> <“computer”, “who is the best football player in Europe to date”> <“finance”, “who is the best football player in Europe to date”>

For model training, we input one-to-one tuples that correspond to the text and label dictionary and output predictions labeled TRUE/FALSE.

We provide ALBERT with additional class label text input. This requires ALBERT to understand the connection between class labels and questions. We use sentence fragments [29] to represent class labels and questions; we use ALBERT's special separator token [SEP] to add class labels to the text. Since the input of ALBERT can be a single sentence or a set of sentence pairs, as seen in Figure 2, to preset the class label to the question, we treat the class label as a sentence. The input text is in the format “[CLS] x1 [SEP] x2 [SEP]”, where x1 represents the class label, x2 represents the question, and [SEP] is used to separate the two inputs. The [CLS] token is placed at the top of the first sentence, and it can be used as a representation of the text classification for subsequent classification tasks. Therefore, the input sequence is composed of the [CLS], the class label, [SEP], the question, [SEP], and some tokens in the random MASK questions.

L-ALBERT-FiT maps question (*t*) to an M-dimensional word embedding vector, where each dimension (i) corresponds to label (*y*_*i*_). A tuple composed of text input is provided, and the class label name corresponds to the (1) function [23] as follows:

(1) $$\begin{array}{c} f:\text{text}⟶{\left\{0,1\right\}}^{M}i.e,f\left(t\right)=P\left(\left.y_{i}\right|t\right)\forall i\in \left\{1\ldots M\right\}\text{.} \end{array}$$

In other words, we provide a tuple of <class labels, question> as the input of L-ALBERT-FiT. The core model architecture of L-ALBERT-FiT is a transformer encoder [18], which includes a multihead attention layer for encoding text, feed-forward layers for calculating nonlinear interlayer features, and layer norms and residuals for deepening the network depth, reducing training difficulty, and performing positional encoding.

### 3.2. Training and Prediction

The backbone of the ALBERT's architecture is the multiheaded, multilayer transformer encoder. The encoder of each layer is composed of a mutihead-attention mechanism and a feed-forward network.

In a transformer, the attention module repeats multiple calculations in parallel. Each of these is called the head attention. Then, this input sequence is passed through all of the head attentions in the ALBERT. The [CLS] token summarizes information from other tokens via the head attention, which facilitates the intrinsic task of pretraining and enabling the [CLS] token to be further optimized while fine-tuning downstream tasks. The representation of the [CLS] token in the final layer is used as a label-dependent representation of the input question.

In Figure 3(a), the transformer encoder converts the inputs into embeddings, and positional encoding obtain the vector *X* from embeddings, input the *X* to the multi-head attention layer. In the multihead attention layer, self-attention helps the current node not only focus on the current word but also obtain the semantics of the context. For the input question, we need to enhance the semantic vector representation for each word separately; therefore, we used each word as a query and weighted the semantic information of all the words to get the enhanced semantic vector for each word. In this case, the vector representations of query, key, and value all come from the same input question, so the attention mechanism of multihead attention layer is also called self-attention. First, self-attention learns a weight for each word of the input vector *X*, maps it to the query (*Q*), key (*K*), and value (*V*) vector, and then calculates a weighted feature matrix by scaled dot-product attention in Figure 3(b), as follows [18]:

(2) $$\begin{array}{c} \text{Attention}\left(Q,K,V\right)=softmax\left(\frac{QK^{T}}{\sqrt{d_{k}}}\right)V\text{,} \end{array}$$

where the input dimensions of key and value are *d*_*K*_and *d*_*V*_. In order to stabilize the gradient, the transformer uses score normalization, which is divided by $\sqrt{d_{k}}$, and the softmax activation function to obtain the weight of the value. As shown in Figure 3(b), the multihead attention means that the self-attention is repeatedly calculated *h* times in parallel. Finally, *h* heads can obtain *h* attention pooling outputs, concat them together, and pass a linear mapping (*W*^*O*^) again to obtain the final output [18] as follows:

(3) $$\begin{array}{c} \text{MultiHead}\left(Q,K,V\right)=\text{Concat}\left({\text{ head }}_{1},\ldots ,{\text{ head }}_{h}\right)W^{O}\text{,}\\ {\text{ where head }}_{i}=\text{Attention}\left(QW_{i}^{Q},KW_{i}^{K},VW_{i}^{V}\right)\text{.} \end{array}$$

Parameter matrices are *W*_*i*_^*Q*^ ∈ *R*^*d*_mo de l_×*d*_*K*_^, *W*_*i*_^*K*^ ∈ *R*^*d*_mo de l_×*d*_*K*_^, *W*_*i*_^*v*^ ∈ *R*^*d*_mo de l_×*d*_*V*_^ and *W*^*O*^ ∈ R^*h* *d*_*V*_×*d*_mo de l_^. All sublayers in the model and the embedding layer produce a dimensionality output as *d*_mo de l_. Then, the refined vector obtained by multihead attention is projected to a higher-dimensional space through the feed-forward layer, making it easier to extract the desired information.

As seen in the previous description, when many embeddings are input, the output has the same number of embeddings; then, we can call the output a hidden vector. When performing a specific NLP task, we only need to take the corresponding hidden vector as the output. The advantage of this is that multiple groups can be calculated in parallel, and different groups can capture information in different subspaces.

Finally, we use the softmax function to form a probability distribution divided into two categories, namely, TRUE/FALSE. We use TRUE/FALSE to replace ALBERT's linear layer, assuming that the *ith* label *y*_*i*_ is the true value of the *jth* question *t*_*j*_ label, then the output is (<label(*y*_*i*_), *t*_*j*_>, TRUE), otherwise, the output is (<label(*y*_*i*_), *t*_*j*_>, FALSE) to train the predictability of the model. Assuming that there are *M* class labels in the class label dictionary, we fill in all of the possible tuples and obtain the TRUE/FALSE prediction of *M* groups through the L-ALBERT-FiT model as follows:

(4) $$\begin{array}{c} \hat{y}=\underset{k\in 1\ldots M}{argmax}\left(\text{label}\left(y_{i}\right),x\right)\text{.} \end{array}$$

If the label matches the question, the output is true; otherwise, the output is false. Each output corresponds to a label, and the prediction result is as follows: < “sports”, “who is the best football player in Europe to date” > -> TRUE. < “relationships”, “who is the best football player in Europe to date”> -> FALSE. < “computer”, “who is the best football player in Europe to date”> -> FALSE. < “finance”, “who is the best football player in Europe to date”> -> FALSE.

The model obtains the semantic information of all of the category labels in the label dictionary, compares the weights of the labels and questions, and calculates the semantic similarity of the two to obtain the relevance of the two. Then, when this classifier is extended to the target domain for classification, on the premise that we know the semantic information of the labels in the target domain, we can predict the similarity based on the weight of the question and the label.

## 4. Experiment Results and Discussion

### 4.1. Experimental Setup

Our model adopts the Flair framework with 12 repeated layers, the initial word embedding dimension is 128, the hidden dimension is 768, the attention-head is 12, and the parameter size is 11 M. The mini batch size is 1, the maximum number of epochs is 15, and each batch is performed for 110 iterations. We use a maximum batch size of 4 to update the parameters. We used the Adam optimizer to optimize the objective function with an initial learning rate of 0.001.

### 4.2. Experimental Data

The dataset is the Yahoo! Answers dataset [30]. The fields of this dataset include question title, question content, and best answer. The title has 10 categories (Society and Culture, Science and Mathematics, Health, Education and Reference, Computers and Internet, Sports, Business and Finance, Entertainment and Music, Family and Relationships, Politics and Government), each category contains 140,000 training samples and 5,000 test samples, and the dataset itself contains more than 4 million Q&A pairs. We divide the dataset into 5 different domains by different category labels, each containing two categories of questions.

We artificially set the source domain and the target domain. The source domain is used to train models and the target domain is used for testing and evaluation. We experiment with different models on different domains, including employing A as the source domain and B as the target domain for cross-domain question classification. Each model performs 5 sets of classification experiments. We randomly select 5000 source domain data points as the training set, 500 source domain data points as the development set (used by some models), and 2000 target domain data points as the test set.

### 4.3. Evaluation Index

The effectiveness of the proposed method is measured by calculating the following metrics: accuracy, which are the most common metrics measurement in question classification. We measure the question classification performance by the accuracy values defined as follows:

(5) $$\begin{array}{c} \text{accuracy}=\frac{\#\;Correctly\;classifie\;d\;questions\;}{\#\;Total\;number\;of\;questions}\text{.} \end{array}$$

### 4.4. Method and Results

#### 4.4.1. Traditional Nontransfer Machine Learning for Cross-Domain Question Classification

In 1998, support vector machines (SVM) [31] were a binary classification model that was a discriminant classifier formally defined by the separated hyperplane. In other words, given labeled training data (supervised learning), the algorithm output an optimal hyperplane to classify new examples. Its basic model was defined as the linear classifier with the largest interval in the feature space, and its learning strategy was to maximize the interval, which could eventually be converted into the solution of a convex quadratic programming problem.

In 1967, Cover and Hart formally introduced the K-nearest neighbor (KNN) algorithm [32], and KNN was a nonparametric supervised classification model. It could assign labels based on calculating the distance from *k* training samples to the query point. In the classification stage, *k* was a user-defined constant. A vector without category labels (query or test point) would be classified as the most frequently used class of the *k* sample points closest to the point.

Thomas Bayes proposed Bayes' theorem [33], which describes the probability of an event based on prior knowledge of the event. This can be calculated as follows:

(6) $$\begin{array}{c} P\left(\left.A\right|B\right)=\frac{P\left(A\cap B\right)}{P\left(B\right)}=\frac{P\left(A\right)\cdot P\left(\left.B\right|A\right)}{P\left(B\right)}\text{.} \end{array}$$

It is assumed that the occurrence of each word in the text is independent. The text classification problem based on such assumptions can be solved by the naive Bayes method.

Table 1lists the accuracy of three traditional machine learning classifiers that directly perform question classification in the target domain after the source domain training is completed (%, keep 2 digits after the decimal point). Among these, AVG-T represents the average classification accuracy%. We took 5,000 questions from each domain and performed the experiments as the training set (source domain) and the test set (target domain).

Traditional question classification methods do not use transfer learning and directly use the source domain-trained classifier to classify the target domain questions. As seen from Table 2, SVM, Bayes, and KNN have poor classification effects on the target domain, and the average accuracy is only 57.24%, far from meeting the requirements of cross-domain question classification.

#### 4.4.2. Transfer Learning Cross-Domain Question Classification

To assess the ability of nontransfer versus transfer learning in different domains, we perform the following experiments. We report the classification accuracy of different transfer schemes on target domains. Under the above experimental conditions, we perform cross-domain question classification experiments on several common traditional transfer learning models and deep transfer learning models, while the model parameters restore the settings in their baseline articles when the number of JDA iterations is set to 15.

Table 3 lists the accuracies of the 2 traditional and 5 deep transfer models on cross-domain question classification (retaining the top 2 after the decimal point). Among them, AVG-T represents the average classification accuracy rate of the traditional classifier. AVG-TT represents the average classification accuracy rate of the traditional transfer classifier. AVG-DT represents the average classification accuracy rate of the deep transfer classifier.

As seen in Figure 4, the nontransfer machine learning classifier performs the worst in the 4 sets of classification experiments, and the traditional transfer classifier is slightly better. In the experiment with source domain B and target domain *E*, the opposite is true, indicating that the improvement of question classification accuracy in a traditional transfer is limited. When the semantic distances of the source domain and the target domain are close, a traditional transfer cannot continue to bring better improvement effects to question classification. Compared with the traditional transfer model, the deep transfer classifier has an average increase of 13.39 percentage points, and the experimental results are stable, which has a considerable improvement effect in different group experiments. Therefore, we can conclude that the application of transfer learning effectively improves the accuracy of cross-domain question classification.

Figure 5 visually reflects the question classification effect of different deep transfer learning classification models on our dataset. According to Figure 5, the BERT and ALBERT models have the highest accuracy in question classification and similar results, while BERT's effect is slightly better than ALBERT's. However, Lan et al. [20] compared the performance of the BERT and ALBERT models of different scales in different NLP downstream tasks. Even though the parameter amount of the ALBERT-xxlarge is much smaller than that of the BERT-large, and ALBERT's F-score gradually increases as the scale increases. As the BERT model increases, this causes the return of NLP to degrade. It is concluded that ALBERT is faster and more effective than BERT when using fewer parameters.

### 4.5. L-ALBERT-FiT

The experiments use the Flair framework with 12 repeat layers, embedding dimensions of 128, hidden dimensions of 768, attention heads of 12, and 11 M parameters. The maximum number of epochs is 20, and each batch performs 110 iterations. We use the max batch size of 4 to update the parameters to optimize the objective function.

We compare L-ALBERT-FiT with the following two baselines:

- BERT-BASE-V2: we pretrain and fine-tune the pretrained BERT model according to the above datasets and test the model in the target domain.
- ALBERT-BASE-V2: it is a BERT variant, which we similarly pretrain and fine-tune, before testing the model in the target domain.

To compare the performance of the model itself, we select the average of 10 experiments.

The classification performance of L-ALBERT-FiT fluctuates in different domains, which may be related to the similarity between different domains and the number of features extracted, but the overall experimental results are improved. In Table 4, we can see that compared with the ALBERT-fine-tune model, the accuracy rate of L-ALBERT-FiT is improved by approximately 6%, which is approximately 3.7% higher than that of BERT-fine-tune. Intuitively, L-ALBERT-FiT improves cross-domain question classifications.

Learning rates (lr) are perhaps the most important hyper-parameters to tune for training neural networks. We also experimented the classification effect of L-ALBERT-FiT transferred from source domain A to target domain B with different learning rates and then detailed the impact of lr on model performance. The experiment was performed for 15 epochs, and the experimental results are listed in Table 5.

Figure 6 shows the convergence of the loss function when lr=0.001 and lr=0.01.  Figure 6(b) represents that the loss converges quickly and drops to a very low value when lr＞0.01, so it is speculated that the model may be in a state of overfitting. However, the loss converges tend to be smooth when the learning rate is 0.001.

It shows that when the initial learning rate is lower than 0.001, the training accuracy of the model is low, indicating that the model has not been trained and the model is underfitting. When the learning rate is greater than 0.001, the learning rate is too large, the loss convergence speed is fast and decreases very low, and the test accuracy rate is reduced. At this time, the model may be overfitting. Therefore, we chose lr=0.001 as the learning rate of the model.

### 4.6. Text Expansion

As a short text, questions contain fewer keywords, and the extracted features are limited, which is not conducive to NLP downstream tasks. Traditional NLP data augmentation [34–36] techniques include synonym substitution, back translation, text surface conversion, noise addition, and cross-expansion methods, which are dedicated to allowing machines to automatically generate text data and obtain more training data. Zhang and Li [37] introduced a federal initialization stage to keep similar data structures in distributed feature extractions, and a federated communication stage is further implemented using deep adversarial learning. In the data feature extraction stage, the word volume of each question in the dataset is expanded without changing the meaning of the question, enabling the model to extract more text features, thereby improving the classification accuracy.

Considering the characteristics of short text, increasing the number of data items does not meet the training objective, so we expand each piece of data. We randomly select 50% of the words except stop words in the question as the core words, then randomly select a synonym [38] corresponding to the core word from WordNet [39], and insert random positions in the original sentence with the augmented sentence.

As seen in Table 6, the meaning of the expanded question does not change, but the length of each question is increased. We use the above preprocessed dataset to train on the L-ALBERT-FiT model, and the experimental results are obtained.

It can be seen in the above table that text expansion in the 4 experimental groups makes a considerable improvement in the classification effect of the target domain, indicating that inserting synonyms in the question can effectively expand the length of the text and extract more features, thus achieving a better classification effect.

The principle of L-ALBERT-FiT is to compare the similarity between the word embedding of the input question and the word embedding of the category label. The core words and question categories are highly related, but the importance of the same word is different for different categories of questions. Therefore, the synonym expansion of questions can increase the similarity between questions and labels.

For example, the core word of the question “what makes friendship click does spark keep going” before expansion is “friendship,” and the category label of the question is “relationship.” After the text is expanded, the question becomes “what makes friendship click make how does perish make the die spark keep friendly relationship going,” core words such as “relationship” and “friendly” are added. At this time, the core words of the question are closer to the label, and the similarity is higher, so the classification accuracy is higher in Table 7.

Beyond that, this method introduces a certain amount of noise to prevent overfitting, and expanding the synonym to the source domain, the model can be well extended to arbitrary unseen target domains.

However, in the experiment with source domain B and target domain *E*, the accuracy does not increase; it decreases probably because the model has achieved an extremely high accuracy in the experimental group and may introduce some interference if the text is extended. For example, the possible polysemy problem of the core word, which causes the question to introduce ambiguous information, or the noise of WordNet itself when the question inserts the near sense word, interferes with the prediction of the model.

Due to the polysemy problem of the core word, for long text, core words undertake contextual context as high-frequency words, which can greatly avoid interference due to ambiguity. However, long texts are not better for predicting than short texts. In this experiment, we extract the label information as input, which makes the core word of each question only belong to one category in theory, but in the real environment under these circumstances, noise interference is inevitable.

Therefore, we conclude that when the classification accuracy rate is relatively low, the introduction of synonyms has a considerable improvement effect on the cross-domain classification accuracy, and if the accuracy has reached a high value, the noise caused by text expansion will instead reduce the classification accuracy.

## 5. Conclusions

In this article, we verify the effect of transfer learning on cross-domain question classification and propose a deep transfer learning cross-domain question classification method that extracts the semantic information of class labels, which achieves strong classification results. Entering one-to-one tuples of all labels and questions when training their similarity to labels causes a problem; the model greatly increases the amount of input data and increases the computational cost. When the target domain categories are unevenly distributed, the experimental recall is low, and the model performs poorly, which may be caused by ALBERT due to internal parameter sharing. Moreover, due to environmental conditions, we use the ALBERT-base-v2 version in the experiment, and currently, there is a larger ALBERT model version, as well as a version for the Chinese NLP task. Future work will begin to solve the problem with computational load and model instability to further improve the experiment. In addition, we will use a larger-scale ALBERT model to further improve the model's reasoning ability and classification effect.

## Figures and Tables

**Figure 1:** A macro flow chart of the training, transferring, and testing processes of the L-ALBERT-FiT model.

**Figure 2:** L-ALBERT-FiT architecture.

**Figure 3:** (a) Transformer-encoder architecture. (b) Multihead attention architecture.

**Figure 4:** The average classification accuracy of multiple nontransfer machine learning, transfer learning, and deep transfer learning classification models in the above 5 sets of cross-domain question classification experiments.

**Figure 5:** The classification accuracy of multiple deep transfer learning classification models in the above 5 sets of cross-domain question classification experiments.

**Figure 6:** Convergence of loss as epoch increases under different learning rates. (a) Learning rate = 0.001. (b) Learning rate = 0.01.

**Table 1:** The accuracy of the traditional nontransfer machine learning classifier in the target domain question classification (%).

Model	A->B	A->C	A->D	B->E	B->A	AVG
SVM	49.94	50.62	53.92	76.88	60.32	58.34
KNN	50.52	51.60	45.36	77.48	50.26	55.04
Bayes	53.02	54.94	48.22	78.44	57.08	58.34
AVG-T	51.16	52.39	49.17	77.60	55.89	57.24

**Table 2:** The domain division of the experimental dataset.

Domain	Category 1	Category 2
A	Society	Science
B	Computers	Business
C	Health	Politics
D	Education	Entertainment
E	Sports	Relationships

**Table 3:** The accuracy of the transfer learning classifier in the target domain question classification (%).

Model		A->B	A->C	A->D	B->E	B->A	AVG
AVG-T		51.16	52.39	49.17	77.60	55.89	57.24

Traditional transfer	TCA	55.02	51.42	49.02	75.36	57.14	57.59
	JDA	55.44	55.00	49.28	73.60	63.76	59.42

AVG-TT		55.23	53.21	49.15	74.48	60.45	58.50

Deep transfer	ULMFIT	63.68	63.66	52.50	83.58	66.14	65.91
	Flair	64.74	58.81	56.52	87.44	61.63	65.83
	XLNet	74.80	71.90	64.20	87.30	70.90	73.82
	BERT	77.30	77.20	68.40	92.40	74.90	78.04
	ALBERT	73.64	77.08	65.62	90.70	72.21	75.85
AVG-DT		70.83	69.73	61.45	88.28	69.16	71.89

**Table 4:** The accuracy of L-ALBERT-FiT, ALBERT-fine-tune, and BERT-fine-tune in cross-domain question classification (%).

Model	A->B	A->C	A->D	B->E	B->A	AVG
BERT-FiT	77.30	77.20	68.40	92.40	74.90	78.04
ALBERT-FiT	73.64	77.08	65.62	90.70	72.21	75.85
L-ALBERT-FiT	80.76	81.68	72.08	95.56	78.77	81.77

**Table 5:** The accuracy of L-ALBERT-FiT, ALBERT-fine-tune, and BERT-fine-tune in cross-domain question classification (%).

Learning rate	Train acc. (%)	Test acc. (%)
0.0001	93.73	67.18
0.0003	92.23	80.16
0.0005	87.11	84.7
0.0007	93.05	81.26
0.001	94.68	80.76
0.005	94.1	74.88
0.01	93.66	77.76
0.02	91.82	68.84

**Table 6:** Contrast before and after expansion of the question text.

Category label	Before text expansion	After text expansion
Relationships	What makes friendship click does spark keep going	What makes friendship click make how does perish make the die spark keep friendly relationship going

Computer	How download road runner custom browser software father stubborn call support	Reciprocal comprise how do unregenerate *i* download road runner hoosier state incorporate custom browser software my father unregenerate in law is stubborn he begetter won *t* incorporate call comprise support

Entertainment	What best old school song ever created must 1994 earlier	What is the mustiness best old school strike rap mustiness song ever created strike civilize must be chance on strike and earlier

**Table 7:** Accuracy (%) for cross-domain question classification on the L-ALBERT-FiT model before and after dataset expansion.

Model	A->B	A->C	A->D	B->E	B->A
Before expansion	80.76	81.68	72.08	95.56	78.77
After expansion	87.95	90.50	80.25	94.55	80.11

## Data Availability

The data used to support the findings of this study are included within the article [30]. The Yahoo! Answers dataset can be derived from the URL (https://www.kaggle.com/soumikrakshit/yahoo-answers-dataset).
